The article "Identification of the Key Genes Involved in the Effect of Folic Acid on Endothelial Progenitor Cell Transcriptome of Patients with Type 1 Diabetes" was published in 2020. Journal: Comput Math Methods Med.

# Identification of the Key Genes Involved in the Effect of Folic Acid on Endothelial Progenitor Cell Transcriptome of Patients with Type 1 Diabetes

**DOI:** 10.1155/2020/4542689

**Published:** 2020-09-24

**Authors:** Yi Lu, Qianhong Yang, Wei Hu, Jian Dong

**Affiliations:** ^1^Department of Cardiology, Minhang Hospital, Fudan University, 170 Xin-Song Road, Shanghai 201199, China; ^2^Department of Geriatrics, Minhang Hospital, Fudan University, 170 Xin-Song Road, Shanghai 201199, China

## Abstract

Type 1 diabetes (T1D) is one of the most common autoimmune diseases in children. Previous studies have suggested that endothelial progenitor cells (EPCs) might be engaged in the regulating of the biological processes in T1D and folic acid (FA) might be engaged in regulating EPC function. The present study has identified 716 downregulated genes and 617 upregulated genes in T1D EPC cases after treated with FA. Bioinformatics analysis has shown that these DEGs were engaged in regulating metabolic processes, cell proliferation-related processes, bone marrow development, cell adhesion, platelet degranulation, and cellular response to growth factor stimulus. Furthermore, we have conducted and identified hub PPI networks. Importantly, we have identified 6 upregulated genes (POLR2A, BDNF, CDC27, LTN1, RAB1A, and CUL2) and 8 downregulated genes (SHC1, GRIN2B, TTN, GNAL, GNB2, PTK2, TF, and TLR9) as key regulators involved in the effect of FA on endothelial progenitor cell transcriptome of patients with T1D. We think that this study could provide novel information to understand the roles of FA in regulating EPCs of T1D patients.

## 1. Introduction

Type 1 diabetes (T1D) belongs to a type of autoimmune diseases featuring the destruction of insulin-producing pancreatic *β*-cells caused by the immune systems [1]. Type 1 diabetes is regarded as one of the most frequent chronic diseases in children and teenagers. It has contributed to a series of symptoms [2]. Insufficient control of hyperglycemia can help develop diabetic nephropathy, neuropathy, and retinopathy, which are the major causes of kidney failure, blindness, and nontraumatic amputation [3]. Patients suffering from T1D are insulin dependent and highly prone to develop vascular diseases, end-stage renal disease, and neurological damages [3]. The detailed mechanisms regulating T1D and novel therapeutic strategies for this disease remain to be further explored. Endothelial progenitor cells (EPCs) stem from the bone marrow and are critical in regulating revascularization and endothelial homeostasis [3]. Increasing evidence has shown that EPCs are significantly decreased in diabetes patients compared with normal samples, suggesting that EPCs may be involved in the regulating of the biological processes in T1D [4].

The article "Identification of the Key Genes Involved in the Effect of Folic Acid on Endothelial Progenitor Cell Transcriptome of Patients with Type 1 Diabetes" was published in 2020. Journal: Comput Math Methods Med.

With the development of RNA-sequence and microarray methods, emerging studies have explored the pathological mechanisms of human diseases using these novel methods and a lot of data are produced. By analyzing the big data, the researchers could find novel and useful information to understand the progression of human diseases. For example, Safari et al. have reported that YBX1, SRPK1, PSMA1/3, and XRCC6 were key regulators of T1D by using protein-protein interaction network analysis. Jia et al. have identified 329 downregulated genes and 192 upregulated genes in childhood-onset type 2 diabetes [5]. Van et al. have reported that against healthy subjects, there were 1591 genes differently expressed in T1D samples [6].

Folic acid (FA) has been reported to be important in human cell proliferation [7]. Several previous studies have shown that FA was involved in regulating endothelial progenitor cell function and associated with the progression of coronary artery disease, hypercholesterolemia, and diabetes. However, the mechanisms of FA in regulating T1D remain unclear. This study has tried to determine differentially expressed mRNAs after treated with FA by analyzing a public dataset (GSE17635) [8]. Furthermore, coexpression analysis and bioinformatics analysis have been used to identify hub genes involved in the effect of FA on endothelial progenitor cell transcriptome of patients with T1D.

## 2. Material and Methods

### 2.1. Microarray Data

The microarray data of GSE17635 are accessible in the National Center of Biotechnology Information (NCBI) Gene Expression Omnibus database (GEO, http://www.ncbi.nlm.nih.gov/geo/). This dataset is aimed at investigating the difference between the gene expression profiles of endothelial progenitor cells from T1D patients before (*n* = 11) and after a four-week duration of FA supplementation (*n* = 10) and that from healthy subjects (*n* = 11). Patients with T1D (*n* = 20) were diagnosed no less than one year prior to the participation in this study. They were all from the outpatient clinic of the Department of Internal Medicine of the University Medical Centre Utrecht, The Netherlands. In manifest liver disease, macrovascular disease, creatinine > 120 *μ*mol/L, homocysteine > 15 *μ*mol/L, and untreated thyroid disease, the exclusion criteria were present. If those patients were receiving retreatment of vasoactive medication (angiotensin II antagonists, angiotensin-converting enzyme inhibitors, nonsteroidal anti-inflammatory drugs (NSAIDs), statins, vitamins, or FA), then the treatment ceased no less than three weeks before starting this study. Twenty both age-matched and gender-matched participants who were in healthy conditions acted as controls. A questionnaire was used to appraise the cardiovascular risk, and the measurement of some clinical parameters like blood pressure, length and weight was carried out.

The article "Identification of the Key Genes Involved in the Effect of Folic Acid on Endothelial Progenitor Cell Transcriptome of Patients with Type 1 Diabetes" was published in 2020. Journal: Comput Math Methods Med.

The collection of the peripheral blood samples from twenty subjects with T1D and twenty age-matched and gender-matched healthy controls (CTR) at baseline was conducted. A 4-week treatment with FA (Ratiopharm) 5 mg/day was served to T1D subjects, and then, the collection of peripheral blood samples (19/20 patients) was conducted again. The protocol of this study has obtained approval from the Medical Ethical Committee of the University Medical Centre Utrecht. The written informed consent [9] has been provided by all the participants in this study.

GEO provided the downloads of the original datasets, and the log2 transformation was employed to preprocess them. The use of the limma package in R software version 3.3.0 (https://www.r-project.org/) has helped normalize all the sample data. By employing the linear models for microarray analysis (Limma) method [10], the identification of the differentially expressed mRNA and lncRNAs was achieved. An unpaired *t*-test was employed to count the *P* value of each gene, and the Benjamini-Hochberg (BH) method [11] was employed to adjust the *P* value into a false discovery rate (FDR). Only those genes, the FDR of which was less than 0.01, were selected as DEGs.

### 2.2. Construction of the PPI Network and the Module Analysis

As the protein interactions (physical and functional associations) were to be predicted, this study constructed the PPI network for DEGs (the minimum required interaction score > 0.4) [9] employing the Search Tool for the Retrieval of Interacting Genes (STRING). Following this construction of the PPI network, the Mcode plugin (degree cut − off ≥ 2 and the nodes with edges ≥ 2 core) [12] was employed to conduct a module analysis of the network. Besides, in order to visualize the PPI networks [11], Cytoscape software version 3.4.0 (http://cytoscape.org/download_old_versions.html) was employed.

### 2.3. GO and KEGG Pathway Analyses

To figure out how DEGs function, this study has used DAVID system [13] (https://david.ncifcrf.gov/tools.jsp) to perform the analysis of the GO function enrichment and the KEGG pathway enrichment. The *P* value (hypergeometric *P* value) denotes the significance of the pathway associated with the conditions. *P* < 0.05 was considered to indicate a statistically significant difference.

## 3. Results

### 3.1. Identification of DEGs in EPC of T1D Patients after Treated with FA

This study has conducted the analysis of a public expression profiling (GSE17635) in order to determine differently expressed genes (DEG) in endothelial progenitor cells after treated with PA. This dataset has included a total of 11 non-treated T1D EPC samples and 10 PA treated T1D EPC samples. This study has shown that 617 genes were overexpressed and 716 genes were downregulated in T1D EPC samples after treated with PA. Hierarchical clustering analysis of the DEGs is presented in Figure 1. The top 10 upregulated and downregulated genes after FA treatment were shown in Table 1.

The article "Identification of the Key Genes Involved in the Effect of Folic Acid on Endothelial Progenitor Cell Transcriptome of Patients with Type 1 Diabetes" was published in 2020. Journal: Comput Math Methods Med.

### 3.2. Functional Annotation of DEGs in EPC of T1D Patients after Treated with FA

Furthermore, in Figure 2, we have performed GO analysis for these DEGs. Bioinformatics analysis has shown that upregulated genes were related to the regulation of a smoothened signaling pathway, ventricular system development, negative regulation of cell growth, meiotic cell cycle, very long-chain fatty acid metabolic process, collateral sprouting, glycosaminoglycan metabolic process, bone marrow development, response to pain, and ER to Golgi vesicle-mediated transport.

Meanwhile, this study has also shown that downregulated genes were associated with the regulation of positive regulation of transcription from RNA polymerase I promoter, homophilic cell adhesion via plasma membrane adhesion molecules, cell-cell signaling, cell adhesion, embryonic skeletal system development, platelet degranulation, organ morphogenesis, cellular response to growth factor stimulus, regulation of potassium ion transport, and ion transmembrane transport.

### 3.3. PPI Network Analysis of DEGs

The prediction of the interaction relationship between 617 upregulated DEGs and 716 downregulated DEGs has been achieved by using the STRING database. This study first sets up the PPI network by the use of these DEGs. After constructing the PPI network, the Mcode plugin (degree cut − off ≥ 3 and the nodes with edges ≥ 3 core) was employed to carry out a module analysis of it. The identification of 23 hub-networks was found in the downregulated DEG-mediated PPI networks and that of 17 hub-networks in the upregulated DEG-mediated PPI networks.

Figure 3 has presented the top 3 hub-networks in upregulated DEG-mediated PPI networks.  Figure 3(a) shows that there are 18 nodes and 183 edges in Hub-network 1.  Figure 3(b) shows that there are 35 nodes and 142 edges in Hub-network 2.  Figure 3(c) shows that there are includes 37 nodes and 94 edges hub-network 3. Six DEGs, including POLR2A, BDNF, CDC27, LTN1, RAB1A, and CUL2, have been identified as key upregulated regulators by interacting with more than 20 DEGs.

Figure 4 has presented the top 3 hub-networks in downregulated DEG-mediated PPI networks.  Figure 4(a) makes it clear that 13 nodes and 78 edges exist in Hub-network 1.  Figure 4(b) makes it clear that 8 nodes and 28 edges exist in Hub-network 2.  Figure 4(c) makes it clear that 15 nodes and 49 edges exist in Hub-network 3. Eight DEGs, including SHC1, GRIN2B, TTN, GNAL, GNB2, PTK2, TF, and TLR9, have been identified as key downregulated regulators by interacting with more than 20 DEGs.

The article "Identification of the Key Genes Involved in the Effect of Folic Acid on Endothelial Progenitor Cell Transcriptome of Patients with Type 1 Diabetes" was published in 2020. Journal: Comput Math Methods Med.

## 4. Discussion

Endothelial progenitor cells (EPCs) are critical in regulating the revascularization and endothelial homeostasis. Increasing evidence has shown that EPCs were notably decreased in diabetes patients compared with normal samples, suggesting that EPCs might be involved in the regulating of the biological processes in T1D. FA has been reported to act significantly in human cell proliferation. Several previous studies have shown that FA was involved in regulating endothelial progenitor cell function and associated with the progression of diabetes. For example, Anna et al. have reported that metabolic control in overweight T1D patients can be improved through DCI plus FA oral supplementation [14]. Alian et al. have found that FA administration decreased the level of endothelial dysfunction measured [15]. However, the mechanisms of FA in regulating T1D remain unclear. This study has identified DEGs involved in endothelial progenitor cells after treated with FA. The present study has also discovered that 617 genes were overexpressed and 716 genes were downregulated in T1D EPC samples after treated with FA. Furthermore, in order to identify hub genes, two PPI networks have been constructed.

Moreover, we have conducted the bioinformatics analysis for these DEGs in T1D. Our results have shown the involvement of upregulated genes in regulating multiple metabolic and cell proliferation processes, such as cell cycle and very long-chain fatty acid metabolic process. The study has also shown that these DEGs were associated with bone marrow development, which may be modulated by EPC cells. Meanwhile, this study has suggested that downregulated DEGs were involved in regulating cell adhesion, platelet degranulation, and cellular response to growth factor stimulus. These growth factors had been demonstrated to have a crucial role in T1D disease progression. For example, insulin-like growth factor-1 activates AMPK to augment mitochondrial function and correct neuronal metabolism in sensory neurons in type 1 diabetes [16]. Fibroblast growth factor 21 ameliorates diabetes-induced endothelial dysfunction in mouse aorta via activation of the CaMKK2/AMPK*α* signaling pathway [17]. Inhibition of epidermal growth factor receptor activation is associated with improved diabetic nephropathy in type 2 diabetes [18].

The article "Identification of the Key Genes Involved in the Effect of Folic Acid on Endothelial Progenitor Cell Transcriptome of Patients with Type 1 Diabetes" was published in 2020. Journal: Comput Math Methods Med.

By conducting PPI network analysis, we have identified 3 downregulated hub-networks and 3 upregulated hub-networks involved in the effect of FA on endothelial progenitor cell transcriptome of patients with T1D. Importantly, we have identified 6 upregulated genes (POLR2A, BDNF, CDC27, LTN1, RAB1A, and CUL2) and 8 downregulated genes (SHC1, GRIN2B, TTN, GNAL, GNB2, PTK2, TF, and TLR9) as key regulators in this progression. Among these regulators, BDNF has been considered to be linked with the prognosis and progression of diabetes. For instance, the reduction of BDNF is regarded to partly lead to cognitive impairment in type 2 diabetes mellitus (T2DM) [19]. Proteome profiling of mitochondria analysis has shown that RAB1A was upregulated in T2DM. SHC1 has been identified as a key regulator in T1D. In a mouse model of T1D, TLR9 has been found to negatively regulate pancreatic islet beta cell growth and function. These results have suggested that the effect of FA on EPC cells in T1D may depend on these key regulators.

## 5. Conclusion

In conclusion, we have identified 716 downregulated and 617 upregulated genes in T1D EPC cases after treated with FA. Bioinformatics analysis has shown the involvement of these DEGs in regulating metabolic processes, cell proliferation-related processes, bone marrow development, cell adhesion, platelet degranulation, and cellular response to growth factor stimulus. Furthermore, we have conducted and identified hub PPI networks. Importantly, 6 upregulated genes (POLR2A, BDNF, CDC27, LTN1, RAB1A, and CUL2) and 8 downregulated genes (SHC1, GRIN2B, TTN, GNAL, GNB2, PTK2, TF, and TLR9) have been identified as key regulators involved in the effect of FA on endothelial progenitor cell transcriptome of patients with T1D. We think that this study could provide novel information to understand the roles of FA in regulating EPC of T1D patients.

## Figures and Tables

**Figure 1:** Identification of the significantly differentially expressed mRNAs in T1D patients after treated with FA. Heatmaps of the differentially expressed mRNAs in GSE17635, upregulated mRNAs, and downregulated mRNAs between control and treated sample with FA.

**Figure 2:** GO analysis of DEGs in EPC of T1D patients after treated with FA. (a) The analysis of the biological processes of the upregulated expressed mRNAs in EPC of T1D patients by treated with FA. (b) The analysis of the biological processes of the downregulated expressed mRNAs in EPC of T1D patients by treated with FA.

**Figure 3:** Construction of PPI network by upregulated DEGs. The PPI networks of upregulated DEGs in the top 3 hub-networks: (a) 18 nodes, 183 edges in hub-network 1; (b) 35 nodes, 142 edges in hub-network 2; and (c) 37 nodes, 94 edges in hub-network 3.

The article "Identification of the Key Genes Involved in the Effect of Folic Acid on Endothelial Progenitor Cell Transcriptome of Patients with Type 1 Diabetes" was published in 2020. Journal: Comput Math Methods Med.

**Figure 4:** Construction of PPI network by downregulated DEGs. The PPI networks of downregulated DEGs in the top 3 hub-networks: (a) 13 nodes, 78 edges in hub-network 1; (b) 8 nodes, 28 edges in hub-network 2; and (c) 15 nodes, 49 edges in hub-network 3.

**Table 1:** The top 10 upregulated and downregulated genes after FA treatment.

Gene name	*P* value	Ave nontreatment	Ave treatment	Fc	Regulation
TFRC	0.006293	11.00542	12.23194	2.340016	Upregulated
ZFAND5	0.008766	10.48779	11.68049	2.285802	Upregulated
PPA2	0.008097	10.19328	11.31317	2.173302	Upregulated
LIMS1	0.004958	9.447019	10.47183	2.034697	Upregulated
SPTLC1	0.007231	9.948845	10.89993	1.933331	Upregulated
GPR183	0.008343	10.03497	10.92472	1.852857	Upregulated
STRAP	0.006873	9.901829	10.78517	1.844646	Upregulated
XPO1	0.003324	9.896716	10.76951	1.831212	Upregulated
RAB1A	0.002892	11.08631	11.94823	1.81746	Upregulated
UGP2	0.002848	10.00758	10.86298	1.80927	Upregulated
C19orf24	0.008067	11.64242	11.01402	0.646894	Downregulated
PBX2	0.0019	10.39015	9.723368	0.62991	Downregulated
CCDC106	0.007927	10.40376	9.722742	0.623726	Downregulated
SPATA20	0.00734	10.03424	9.332935	0.615015	Downregulated
PPP6R1	3.43E-05	9.85842	9.156729	0.614851	Downregulated
S100A10	0.007334	11.94692	11.22914	0.608032	Downregulated
PDLIM1	0.006748	9.121195	8.402882	0.607808	Downregulated
HVCN1	0.009486	10.39443	9.670834	0.605587	Downregulated
LHPP	0.000472	9.838647	9.111007	0.603891	Downregulated
LTBP2	0.002257	9.206243	8.462812	0.597317	Downregulated
TMEM156	0.008418	10.49832	9.638557	0.551042	Downregulated

## Data Availability

The datasets used and/or analyzed during the current study are available from the corresponding author on reasonable request.
